The article "Lead, Cadmium and Cobalt (Pb, Cd, and Co) Leaching of Glass-Clay Containers by pH Effect of Food" was published in 2011. Journal: Int J Mol Sci.

# Lead, Cadmium and Cobalt (Pb, Cd, and Co) Leaching of Glass-Clay Containers by pH Effect of Food

**DOI:** 10.3390/ijms12042336

**Published:** 2011-04-04

**Authors:** Carmen Valadez-Vega, Clara Zúñiga-Pérez, Samuel Quintanar-Gómez, José A. Morales-González, Eduardo Madrigal-Santillán, José Roberto Villagómez-Ibarra, María Teresa Sumaya-Martínez, Juan Diego García-Paredes

**Affiliations:** 1 Institute of Health Sciences, Autonomous University of Hidalgo State, Ex-Hacienda de la Concepción, Tilcuautla, 42080 Pachuca de Soto, Hgo, Mexico; E-Mails: zupecl@yahoo.com.mx (C.Z.-P.); jmorales101@yahoo.com.mx (J.A.M.-G.); eomsmx@yahoo.com.mx (E.M.-S.); 2 Basic Science and Engineering Institute, Autonomous University of Hidalgo State, Ex-Hacienda de la Concepción, Tilcuautla, 42080 Pachuca de Soto, Hgo, Mexico; E-Mail: Roberto_ibarrav@hotmail.com; 3 Secretary of Research and Graduate Studies, Autonomous University of Nayarit, Ciudad de la Cultura “Amado Nervo”, Blvd. Tepic-Xalisco S/N. Tepic, Nayarit, Mexico; E-Mails: teresumaya@hotmail.com (M.T.S.-M.); digapa1@hotmail.com (J.D.G.-P.)

**Keywords:** leaching, heavy metals, glass clay

## Abstract

Recent studies have shown that handcrafted glass-clay containers are a health risk because they can be contaminated by heavy metals, which can be transferred to food, thus reaching the human body to potentially cause illness. Therefore, in the present work, we evaluate the leaching of lead, cadmium, and cobalt from glass-clay containers into two types of food: tomato sauce (salsa), and chickpea puree. The containers were obtained from four regions in the Mexican state of Hidalgo. Repetitive extractions from the containers were carried out to quantify the leaching of the heavy metals into the salsa, the chickpea puree, and acetic acid using the technique proposed by the USFDA. The results show that greater use of the containers leads to more leaching of heavy metals into both types of food and into the acetic acid, with the greatest metal extraction recorded for the Ixmiquilpan vessels. These results indicate that the metals present in the glass-clay containers leach into the food and that increased reuse increases the risk to the people who use them in food preparation.

## 1. Introduction

The development of technology, large-scale and indiscriminate consumption of fuel, and industrial chemical waste have caused the presence of considerable metal concentrations in the environment, which can exert several different effects on the ecosystem [1,2]. However, the incidence of metals in nature ranges beyond domestic and industrial processes to natural deposits that are found in the Earth’s crust and to a natural presence in the air, water, and soil [3,4]. Regardless of the source of the metals found in the environment, many of them play an important role in all life forms. For example, cobalt, iron, chrome, zinc, and manganese are essential to plants and animals. However, elements such as lead, cadmium, arsenic, beryllium, mercury, and barium have not shown any beneficial function in human beings [5,6].

The article "Lead, Cadmium and Cobalt (Pb, Cd, and Co) Leaching of Glass-Clay Containers by pH Effect of Food" was published in 2011. Journal: Int J Mol Sci.

Although the toxicity of a metal depends on the amount ingested, chronic exposure to certain metals, such as arsenic and lead, can cause severe toxic effects, even in low amounts. Humans are exposed to metals through different exposure pathways, the most common being inhalation of contaminated air and ingestion of products such as water, medicinal herbs, and food [7–10].

Lead is considered to be among the most dangerous metals for human health because it affects the central nervous system, causes anemia and gastrointestinal damage, and is associated with alterations in genetic expression [11–15]. Cadmium is even more dangerous, being 10 times more toxic than lead, and is an element to which humans are readily exposed due to its large industrial use. This metal has been associated with problems in respiratory pathways, including lung cancer [16–18], problems in the gastrointestinal system [19,20], and, although it has shown a very small mutagenic effect, it has been linked with genotoxic effects in some eukaryotic cells, such as in the testicles [21], and with inhibited DNA repair [22,23]. Cobalt is an element that is not easily found in free form in the environment, but is known for being introduced into the food chain due to its absorption by plants in the forms of fertilizers and industrial pollutants [24–26]. Exposure to cobalt can cause damage to respiratory pathways and to the lungs, heart, and thyroid [27–29].

The presence of metals in food can be caused by different sources, such as by direct contamination during production, from metal-rich soil, air, or contaminated water, or from the use of pesticides or fertilizers. Food can also be contaminated during transport, industrial processing, or during storage [30–32]. The domestic preparation of food as a potential source of heavy-metal contamination has been afforded little importance. However, there are reports that indicate that certain kitchen utensils used for food preparation can represent a significant risk because they are manufactured with materials that can be hazardous or contaminated by toxic metals [33–35].

In Mexico and in some other countries, different glass-clay containers are handcrafted and used for the preparation, storage, and consumption of food. By their very nature, these containers can be contaminated with heavy metals, which can derive from the raw materials used in their manufacturing, such as clay, water, and enamel [33,36]. The problem with the presence of heavy metals in glass-clay containers lies in the fact that these contaminants can be transferred to food by a leaching process, which is directly related with the physical and chemical conditions of the food, such as temperature and pH [37,38].

The article "Lead, Cadmium and Cobalt (Pb, Cd, and Co) Leaching of Glass-Clay Containers by pH Effect of Food" was published in 2011. Journal: Int J Mol Sci.

Therefore, sequential leaching of cadmium, cobalt, and lead into food stored in glass-clay vessels from four municipalities of the state of Hidalgo in Mexico is evaluated in the present work.

## 2. Experimental Section

### 2.1. Samples

The clay, the enamel litargirio (termed *greta* by the manufacturers), and 12 glass-clay containers were obtained directly from a sole manufacturer in each locality of the four regions of the state of Hidalgo: Huejutla; Ixmiquilpan; Tepetitlán, and Tulancingo. Samples of the clay and the enamel used in the manufacturing of the containers were also collected.

All containers were washed with detergent and a commercial dish-scrubbing fiber (Scotch Brite), simulating everyday use, rinsed with deionized water, and dried in an oven (Scorpion Scientific, Model D 1754) at a temperature of 25 °C for 24 h [37].

### 2.2. Preparation of Food

Two types of food with different pH were prepared. One consisted of a green tomato sauce traditionally consumed by the population (salsa) based on husk tomato (*Phisalis phyladelphica Lam.*), serrano pepper (*Capsicum frutescens*), garlic (*Allium sativum*), and onion (*Allium cepa*), with a pH of 4.2. The second type of food was a chickpea puree (*Cicer arietinum*) cooked in water, with a pH of 6.0.

### 2.3. Leaching of Heavy Metals into Food

One glass-clay recipient per region was filled with 300 mL of salsa or puree and stored for 24 h at 4 °C. Subsequently, the food was removed, and a 1 g aliquot of each food type was subjected to digestion as described later. The containers were then washed and dried again as previously indicated to simulate the wear and tear that they undergo during frequent use. The containers had the respective food type placed in them again, and the initial conditions were again performed. The entire procedure was repeated a total of 10 times. The test was performed in triplicate for each study area and for each food type; for each repetition of the study regions and food, we employed a new glass-clay container.

### 2.4. Heavy-Metal Leaching Effect in Glass-Clay Containers with Acetic Acid

The heavy-metal leaching technique described by the US Food and Drug Administration (FDA) was used with some modifications, as described González de Mejía *et al.* [37]. The leaching of Cd and Co was followed according to the method established for Pb by the FDA as follows: a new container for each of the four areas studied, previously washed and dried, was filled with 300 mL of acetic acid (4% pH 2.75) and heated to 35 °C for 45 h to simulate the wear of the protective enamel and the leaching of the studied metals in the vessels due to continuous use and reuse. Every 3 h, a 10 mL aliquot of acetic acid was taken until a series of 15 samplings in triplicate per area studied was completed. A 1 mL aliquot of the acetic acid of each sample was taken and digested. The testing was conducted in triplicate for each area, employing a new container on each occasion.

The article "Lead, Cadmium and Cobalt (Pb, Cd, and Co) Leaching of Glass-Clay Containers by pH Effect of Food" was published in 2011. Journal: Int J Mol Sci.

### 2.5. Extraction of Metals in Clays and Enamels Used in the Manufacturing of the Containers

A 1 g aliquot of enamel or clay was taken and digested with dihydrogen peroxide and acetic acid as mentioned later, performing the procedure in triplicate.

### 2.6. Digesting of Samples

The samples obtained in the previously mentioned experiments were digested with 1 mL of hydrogen peroxide (J.T. Baker, Mexico) and 2.5 mL of concentrated nitric acid (J.T. Baker, Mexico) in a Teflon TFM vessel with a Milestone Start D microware digestion system (Multiwave Anton Paar, Perkin-Elmer, Austria) with 75 bars of pressure and 500 watts of power at 280 °C for 35 min. Next, the sample was filtered with 0.4-micron pore-sized Whatman paper and the samples were stored at 4 °C [39].

### 2.7. Quantification of Cd, Co, and Pb

The concentrations of Cd, Co and Pb were determined by inductively coupled plasma spectrometry (ICP/O, Perkin-Elmer Optima 3000 XL, Austria). Measurements were performed for each of the triplicates of leaching tests and for each region under study. The limits of detection were the following: Cd, 0.15 ppb; Co, 3.0 ppb, and Pb, 0.30 ppb. We made a calibration curve using a standard multi-ionic containing Cd, Co, and Pb at concentrations of 0, 0.5, 1.5, 3, 5, and 7 ppm. The accuracy of the instrumental methods and analytical procedures was checked by performing the measurements in triplicate. Analytical-grade reagents (J.T. Baker) were used for the blanks and calibration curves.

### 2.8. Data Analysis

The results were evaluated statistically using the statistical software SPSS 12.0. The two-way ANOVA test was applied to study variance. The statistical significance of the differences was assessed by applying the Tukey test. A probability of 0.05 or lower (*p* ≤ 0.05) was considered significant.

## 3. Results

### 3.1. Quantifying Cd, Co, and Pb in Enamels and Clays Used for the Manufacture of Glass-Clay Containers

Table 1 shows the content of Cd, Co, and Pb present in the enamels utilized in the manufacture of glass-clay vessels. No difference was observed in heavy-metal concentration in the four areas studied. The highest content of Cd and Pb was found in the Huejutla sample, while the highest content of Co was found in the Tulancingo sample.

The article "Lead, Cadmium and Cobalt (Pb, Cd, and Co) Leaching of Glass-Clay Containers by pH Effect of Food" was published in 2011. Journal: Int J Mol Sci.

The Cd, Co, and Pb concentrations in the clays used to manufacture glass-clay containers are shown in Table 2. It can be observed that the concentration of these metals is statistically different in each region studied, with the Ixmiquilpan region having the maximum metal concentrations of 757.99, 571.39, and 833.73 ppm for Cd, Co, and Pb, respectively, whereas Tulancingo had the lowest concentration.

### 3.2. Leaching of Cd, Co, and Pb into Green Tomato Sauce (Salsa) at pH 4.2

Figures 1, 2, and 3 show the Cd, Co, and Pb content due to the leaching of glass-clay containers into green tomato sauce (salsa) for the four regions studied after 10 extractions. It can be observed that the concentration of metals differs in each region studied, with the vessels from Ixmiquilpan having the largest amount of leached Cd, Co, and Pb after 10 extractions. The concentration ranges were 1.33 to 54.12 ppm for Cd, 2.40 to 27.67 ppm for Co, and 5.30 to 63.33 ppm for Pb. On the other hand, the clay containers from the Tulancingo region showed the least amount of leaching of the three metals, in which the concentrations ranged from 0.74 to 16.15 ppm for Cd, from 0.78 to 17.34 ppm for Co, and 1.52 to 28.93 ppm for Pb.

The statistical analysis shows significant differences for each metal among the municipalities studied, with the greatest concentrations of Cd, Co, and Pb found in Ixmiquilpan (54.12, 27.67, and 63.33 ppm, respectively).

### 3.3. Leaching of Cd, Co, and Pb in Chickpea Puree at pH 6.5

Figures 4, 5, and 6 show the Cd, Co, and Pb concentrations caused by the leaching of the glass-clay containers into the chickpea puree in the four regions after 10 extractions. The results show significant differences among the sampling locations and the analyzed metals, with the Ixmiquilpan vessels having the greatest leaching of the three metals. For this region, the Pb levels were the highest (1.97–13.40 ppm), followed by Cd (1.65–11.57 ppm) and Co (1.23–7.03 ppm). The Tulancingo vessels had the lowest levels, ranging between 1.11 and 8.23 ppm for Pb, between 0.7 and 5.73 ppm for Cd, and between 1.39 and 2.48 ppm for Co.

### 3.4. Leaching of Cd, Co, and Pb with Acetic Acid at pH 2.75

The leaching of Cd, Co, and Pb with a series of 15 extractions with acetic acid from the glass-clay containers are shown in Figures 7, 8, and 9. It can be observed that the sampling locations show a statistical difference in the concentrations of leached metals. The Ixmiquilpan vessels have the greatest leached concentrations of the three metals, with levels within the range of 2.24–127.52 ppm for Cd, 2.4–70.38 ppm for Co, and 4.0–188.08 ppm for Pb. On the other hand, the clay containers from Tulancingo have the lowest metal concentrations: Co (0.39–41.46 ppm); Cd (1.43–74.59 ppm), and Pb (2.86–106.52 ppm).

The article "Lead, Cadmium and Cobalt (Pb, Cd, and Co) Leaching of Glass-Clay Containers by pH Effect of Food" was published in 2011. Journal: Int J Mol Sci.

## 4. Discussion

The clays used in the manufacturing of glass-clay containers are very diverse. On occasion, a mixture of clays from different areas is used to obtain an ideal mixture. Therefore, the metal content in the containers depends on the origin of the clays, causing significant variation. These clays have silicon oxide as their main component, as well as other complex silicates, and kaolin, alumina, and feldspar. Due to their nature, they can also have various amounts of different metals. Unfortunately, Mexico does not exert toxicological control over the clays; thus, the final product can have various levels of heavy metals. The natural diversity of each clay lot means that its composition varies considerably, and the containers made from this clay therefore also vary in composition.

As was observed in this work, the Cd, Co, and Pb content in the four analyzed clay samples vary significantly, which is due to the very diverse composition of their sources. The high metal content observed indicates the absence of quality control of this material and makes the need evident for the government to exercise preventive measures in this situation by enforcing the quality control of raw materials such as clay.

For the enamel coating of clay vessels, the craftsmen of the studied regions, as well as in many other regions, employ a product called litharge or *greta*. The results indicate that manufacturers are probably using *greta* from the same company, but it is difficult to know what this is, or what the brands or companies are that provide this type of material, as it is often acquired through intermediaries at low scale.

This product is made from lead oxide, which has benefits to the manufacturers, including low cost and a low melting temperature (<990 °C), rendering it adequate for the manufacturing conditions used by craftsmen and provides the vessels with their characteristic shine. Although the official Mexican code (NOM-231-SSA1-2002) [40] prohibits the use of this type of product in the coating of containers used to store and/or process food or beverages for human consumption, they continue to be used. Their continued use is because people do not know or are ignorant of the law; therefore, materials used for the manufacturing of utensils for human use must not contain lead or any of its derivatives due to the health problems that they cause. The law also states that the use of lead oxide-based enamels, such as litharge, which craftsmen from the studied regions use in the handcraft of clay containers, is not allowed.

The article "Lead, Cadmium and Cobalt (Pb, Cd, and Co) Leaching of Glass-Clay Containers by pH Effect of Food" was published in 2011. Journal: Int J Mol Sci.

The leaching of metals induced by acetic acid, which was used to simulate the prolonged use of the containers, shows that metal leaching increases with increased use of the containers. This method to establish the amount of metals that are leached by acetic acid has been well utilized by several authors [37,41–44], who have shown that clay containers from Mexico, Italy, and other countries have high concentrations of heavy metals, mainly lead, surpassing the limits allowed by the FDA.

Although the use of enamels based on lead or any of its derivatives is prohibited in many countries, such as Mexico, they continue to be used because this type of material is less expensive than their lead-free counterparts, without considering the hazards that they can cause to human health. There are reports [42,45,46] in which a correlation between the use of glass-clay containers covered with lead-based enamel and high blood levels of lead is reported.

Similar to the results of the present work, other researchers [47,48] have observed that the cadmium levels in clay containers can be very high due to the contamination of the raw materials. Both clays and enamels demonstrate high concentrations of this metal, which are leached from the container in greater concentrations the more the container is used, yielding levels above those permitted by the FDA and Mexican law [40].

In our results, the Tulancingo region shows a statistically lower concentration of this metal in food compared with the other regions. However, there is a toxicological risk when the containers are constantly reused because increasing their use degrades the enamel covering the vessel due to acidity and to the friction between the food and the vessel walls, which consequently causes a greater concentration of heavy metals to leach. None of the containers met the limits allowed by Mexican Law for the limits of Cd in glass-clay articles, namely, a permissible maximum of 0.5 ppm. However, the US FDA mandates a maximum cadmium concentration in various ceramic articles of 0.25 ppm, which is why the results of this work show that the studied samples have higher levels of Cd leaching.

Although a permissible limit for the levels of cobalt in the recipients of glass clay has not been officially mandated, it is known that this metal can be toxic to living organisms [49–52]. Therefore, a 1.5 ppm maximum permissible limit of this metal has been reported because higher levels can be related with health problems. As we can see, the levels of Co leached from containers by the acetic acid are higher than the permissible level, beginning with the first extraction and increasing with further container use, reaching concentrations of >70 ppm. Co is essential in trace amounts for living organisms, mainly in the form of vitamin B_12_, and is important for the functioning of red blood cells. Although it is not easily stored in the body, consumption of high amounts can cause adverse effects in lungs, heart, and skin [49–52]. It has also been shown that high amounts of Co can cause severe damage to respiratory pathways, such as degeneration and squamous metaplasia of the olfactory epithelium [29]. Thus, care must be taken with the different exposure pathways for humans because Co levels can increase to levels that pose health risks.

The article "Lead, Cadmium and Cobalt (Pb, Cd, and Co) Leaching of Glass-Clay Containers by pH Effect of Food" was published in 2011. Journal: Int J Mol Sci.

Despite the fact that the lowest levels of leached cadmium and lead were found in Tulancingo, these levels remain higher than those reported by Gould *et al*., in 1983 [41]. However, there are works in which even greater leaching of both metals have been reported [37,42–44].

Similar to the manner in which leaching of metals was observed with acetic acid, release of metals into food was also observed when using two types of food, with pH values of 4.2 and 6.0, with the greater leaching noted with green tomato sauce (salsa), at a pH of 4.2. The effect increased when the clay containers were reused, which agrees with results observed with acetic acid. The results found during the clay vessel re-usage experiments for the leaching of Pb and Cd show that the concentration of heavy metals leached by the clay containers in this study is greater than those reported by Gould *et al*. in 1983 [41] and by González de Mejía *et al.* in 1996 [37]. Several authors ascribe greater importance to metals such as Pb and Cd because these are mainly found in glass-clay containers [37,42–44], affording little importance to metals such as Co because its effects are not as severe as those reported for Cd and Pb.

## 5. Conclusions

The amount of leached metals by chickpea puree, which was at a pH of 6.0, was much less than that observed for acetic acid and green tomato sauce (salsa) at pH 4.2, which indicates that there is a pH dependence on a food’s ability to leach metals, with highly acidic foods causing the greatest leaching of metals from the containers. Based on these results, it is not recommended to use these containers in the preparation and storage of food, even for a short period.

## Figures and Tables

**Figure 1.** Concentration of Cd leached from the glass-clay containers into the green tomato sauce (salsa). The bars show the mean values of the four regions studied with their standard deviations. ^*^ Indicates significant statistical differences with respect to the Ixmiquilpan region, which represents the highest concentration of the metal; *p* ≤ 0.05.

The article "Lead, Cadmium and Cobalt (Pb, Cd, and Co) Leaching of Glass-Clay Containers by pH Effect of Food" was published in 2011. Journal: Int J Mol Sci.

**Figure 2.** Concentration of Co leached from the glass-clay containers into the green tomato sauce (salsa). The bars show the mean values of the four regions studied along with their standard deviations. ^*^ Indicates significant statistical differences with respect to the Ixmiquilpan region, which represents the highest concentration of the metal; *p* ≤ 0.05.

**Figure 3.** Concentration of Pb leached from the glass-clay containers into the green tomato sauce (salsa). The bars show the mean values of the four regions studied along with their standard deviations. ^*^ Indicates significant statistical differences with respect to the Ixmiquilpan region, which represents the highest concentration of the metal; *p* ≤ 0.05.

**Figure 4.** Concentration of Cd leached from the glass-clay containers into the chickpea puree. The bars show the mean values of the four regions with their standard deviations. * Indicates significant statistical differences with respect to the Ixmiquilpan region, which represents the highest concentration of the metal; *p* ≤ 0.05.

**Figure 5.** Concentration of Co leached from the glass-clay containers into the chickpea puree. The bars show the mean values of the four regions along with their standard deviations. * Indicates significant statistical differences with respect to the Ixmiquilpan region, which represents the highest concentration of the metal; *p* ≤ 0.05.

**Figure 6.** Concentration of Pb leached from the glass-clay containers into the chickpea puree. The bars show the mean values of the four regions with their standard deviations. * Indicates significant statistical differences with respect to the Ixmiquilpan region, which represents the highest concentration of the metal; *p* ≤ 0.05.

**Figure 7.** Concentration of leached Cd from the glass-clay containers into acetic acid. The bars show the mean values of the four regions studied, along with their standard deviations. * Indicates significant statistical differences with respect to the Ixmiquilpan region, which represents the highest concentration of the metal; *p* ≤ 0.05.

**Figure 8.** Concentration of Co leached from the glass-clay containers into acetic acid. The bars show the mean values of the four regions with their standard deviations. ^*^ Indicates significant statistical differences with respect to the Ixmiquilpan region, which represents the highest concentration of the metal; *p* ≤ 0.05.

The article "Lead, Cadmium and Cobalt (Pb, Cd, and Co) Leaching of Glass-Clay Containers by pH Effect of Food" was published in 2011. Journal: Int J Mol Sci.

**Figure 9.** Concentration of Pb leached from glass-clay containers into acetic acid. The bars show the mean values of the four regions studied along with their standard deviations. ^*^ Indicates significant statistical differences with respect to the Ixmiquilpan regions, which represents the highest concentration of the metal; *p* ≤ 0.05.

**Table 1.** Cd, Co, and Pb content in enamels used for the manufacturing of glass-clay containers.

**Region**	**Huejutla**	**Ixmiquilpan**	**Tepetitlán**	**Tulancingo**
**Metal**	**Concentration (ppm)**			
Cd	65.95 ± 5.55	63.32 ± 2.90	64.77 ± 0.37	64.46 ± 0.94
Co	43.20 ± 0.45	43.24 ± 1.69	43.20 ± 0.45	44.00 ± 1.98
Pb	64.75 ± 3.05	63.01 ± 3.38	62.60 ± 3.45	63.44 ± 4.20

Mean values ± standard deviation; *p* ≤ 0.05; no significant statistical difference was found among regions.

**Table 2.** Cd, Co, and Pb content in clay used to manufacture glass-clay containers.

**Region**	**Huejutla**	**Ixmiquilpan**	**Tepetitlán**	**Tulancingo**
**Metal**	**Concentration (ppm)**			
Cd	559.56 ± 3.16^a^	757.99 ± 4.16	685.53 ± 7.60^a^	557.99 ± 4.16^a^
Co	472.43 ± 2.77^b^	571.39 ± 3.72	562.82 ± 3.84	468.24 ± 6.18^b^
Pb	621.90 ± 0.52^c^	805.33 ± 1.98	704.40 ± 1.25	607.59 ± 3.48^c^

Mean values ± standard deviation; *p* ≤ 0.05.

Letters indicate significant statistical differences with respect to the region of highest concentration of each metal:

a With respect to Cd;

b with respect to Co;

c with respect to Pb.
